# Indigenous knowledge and quantitative ethnobotany of the Tanawal area, Lesser Western Himalayas, Pakistan

This article has been retracted.

**DOI:** 10.1371/journal.pone.0263604

**Published:** 2022-02-22

**Authors:** Fozia Bibi, Zaheer Abbas, Nidaa Harun, Bushra Perveen, Rainer W. Bussmann

**Affiliations:** 1 Department of Botany, Rawalpindi Women University, Rawalpindi, Pakistan; 2 Division of Science and Technology, Department of Botany, University of Education, Lahore, Pakistan; 3 Department of Botany, Faculty of Life Sciences, University of Okara, Okara, Pakistan; 4 Department of Ethnobotany, Institute of Botany, Ilia State University, Tbilisi, Georgia; Mirpur University of Science and Technology, PAKISTAN

## Abstract

Ethnobotanical field surveys were carried out in the Tanawal area of the Lesser Himalayan Region, Khyber Pakhtunkhawa, Province from April 2016 to October 2017. The area is located between 34.36 (34° 21’ 30 N) latitude and 73.07 (73° 4’ 0 E) longitude with an average elevation of 1374 meters above sea level. Ethnomedicinal data were collected through Participatory Rural Appraisal (PRA), and participants were selected through the snow-boll technique. Semi-structured, in-depth and open-ended interviews were conducted. The data were quantitatively evaluated using ethnomedicinal indices i.e. Relative frequency of citation (RFCs), Fidelity level (FL), and Use Value (UV). The ethnobotanical data were also comparatively analyzed through the Jaccard Index (JI). The study yielded 66 medicinal plants in 62 genera and 43 families. Asteraceae and Solanaceae were the most important families with five medicinal taxa each. Regarding medicinal plant part utilization, leaves (43.28%) were used predominantly, followed by whole plant (14.92%) and fruits (14.92%). Decoction was the main drug formulation applied to 21 species (31.15%) and the oral route was most common (56.1%) while 31.2% of medicinal plants were used for both oral and topical applications. Fifty health disorders were recorded and grouped in 15 categories. Maximum species were used to treat gastrointestinal disorders i.e. 13 species, dermal problems (12 species), and respiratory tract ailments (9). The calculated RFCs ranged between 81 to 31. The most important medicinal plants were *Acacia modesta*, *Citrullus vulgaris*, *Tamarindus indica*, and *Momordica charantia* with an RGFC of 81 each. The UV ranged between 0.58 and 3.6. Medicinal taxa with the highest UV were *Dioscorea deltoidea* (3.6), *Withania coagulans* (3.3), *Momordica charantia* (3.5), *Silybum marianum* and *Pyrus pashia* (3.2). FL values showed that 28 (41.79%) species had a FL value below 50 (74.62%) while 39 (58.20%) had higher FL values. *Momordica charantia*, *Tamarindus indica*, *Acacia modesta* and *Citrullus vulgaris* were 95.2 each. The Jaccard Index (JI) values ranged from16.77 to 0.98. The current study also reported 16 medicinal plants, commonly used around the globe, have been rarely documented for their medicinal values in the local ethnomedicinal literature i.e. *Althaea officinalis*, *Plantanus orientalis*, *Jasminum sombac*, *Maytenus royleana*, *Cucurbita maxima*, *Phyllanthus emblica*, *Citrullus vulgaris*. *Polygonatum verticilliatum*, *Caseria tomentosa*, *Cistanche tubulosa*, *Bambusa arundinacea*, *Schinus molle*, *Tamarindus indica*, *Pongamia pinnata*, *Citrus limon* and *Catharanthus roseus*. However, 48 medicinal plants had been reported in the literature but the current study reported their novel medicinal uses. Important taxa should be established in botanical gardens for in-situ conservation, chemical investigation and sustainable utilization. It would also be effective to improve the livelihoods of the local population.

## Introduction

Mountain landforms are well-known for their biological, geological, climatic, ethnic, cultural and linguistic diversity [1, 2]. They cover 23% of the total global land area and host more than 13% of the global human population. They are also known to be susceptible to different geophysical changes and global climate change [3, 4]. The western part of the Himalayan Mountains located in Khyber Pakhtunkhwa Province of Pakistan includes Kohistan, Mansehra, Abbottabad and Haripur Districts. These occupy lower hilly localities and remote valleys in the high elevations. The area is characterized by moist climate, incredible vegetation and varied topography. Due to these characteristics the territory is also a famous tourist attraction. Presently, these Districts are experiencing escalating human population, increase in tourism infrastructure, developmental projects (roads, dams), efforts of the China Pakistan Economic Corridor (CPEC) and high outmigration trends [5, 6]. Consequently, rapid geo-physical changes can be seen, leading to the displacement of human population, high land-use for construction, destruction of agricultural lands and vegetation. The Pakistan Bureau of Statistics revealed that, based on the 2017census, more than 25 million people with varied ethnic, linguistic and cultural backgrounds reside in these territories (https://www.pbs.gov.pk/). They rely on moist temperate forests for their subsistence, including for fuel wood, fodder, pastures, medicinal plants, timber, and construction materials. The trade of medicinal plants is one the sources of their social livelihoods. Therefore, medicinally important plants often suffer unsustainable utilization, improper collection and bulk extraction [7, 8]. Due to these circumstances the human population and plant based traditional knowledge of the studied area are exposed to a great transition, giving urgency to document and conserve the traditional knowledge of phytotherapies practiced by local people. Fragmented ethnobotanical studies have been conducted in the region of the lesser Himalayas, especially in higher altitude areas, e.g., Abbasi *et al*. (2010), Abbasi *et al*. (2013), Shah *et al*. (2014), Shah *et al*. (2013) and Shah and Khan (2006) [9–13]. The current study site covered various lower hilly and upper sub-alpine localities of the Lesser Himalaya region in the Tanawal area, where no ethnomedicinal study had been conducted yet. We hypothesized that the inhabitants of the study area retain considerable indigenous knowledge of medicinal plants, and used three research questions: 1) how many plants were used as medicine in the studied area? 2) which plants were regarded as highly valued medicinally? 3) how did the medicinal plant knowledge differ from existing regional ethnomedicinal studies?

## Materials and methods

### Study area

Ethnobotanical field surveys were conducted in the Tanawal valley of Khyber Pakhtunkhawa Province from April (2016) to October (2017). The valley is located between the latitude of 34.36 (34° 21’ 30 N) and longitude of 73.07 (73° 4’ 0 E) with an average elevation of 1374 meters above the sea (Fig 1). It is a vast valley and stretches in the areas of three districts i.e. Haripur, Abbottabad, and Mansehra. It borders with Batagram in the north, Tehsil Balakot and Kashmir in the east, a territory of capital Islamabad and Punjab in the south and on the West there are the other districts Swat, Swabi, and Mardan. Geophysically, it is a vast valley and exhibits numerous undulating terraces and hills shaping giving origin to several streams. The rivers Siran and Ichha are the main perennial water bodies. The climate is of the moist temperate type and the region has two rainy seasons: January-February and June- July respectively. The elevated areas are mountainous where snowfall occurs in winter. Floristically the study area falls into the Sino-Japanese regions. The infrastructure is undeveloped and people are still deprived of basic life necessities like electricity, education, and health services. Recently better road connections and communication were established. The population of the area is 315788. People live in small villages along with watercourses. The people are primarily peasants and engaged with small-scale mountain farming.

**Fig 1:** Map of the study area showing villages of three districts; Abbottabad, Mansehra and Haripur.

### Data collection

Consecutive and well-planned field visits of certain 12 sampling sites (Table 1) were made during different seasons in 2016–2017. Before conducting the field surveys, formal written ethical consent was obtained from the local government authorities (Forest departments). Ethnomedicinal data was collected through the Participatory Rural Appraisal (PRA), based on interaction with indigenous people and direct observation in the field [14]. Ethical committee of Rawalpindi Women University and local council of study community provided ethical approval to the study. In addition, before the interviews, verbal prior informed consent was obtained from all respondents. The participants were interviewed by using a semi-structured [15] and an open-ended questionnaire (S1 File). Respondents were selected on the basis of their knowledge, experience and willingness to participate in the study. A total of 85 persons belonging to twelve localities of the three Districts were interviewed in their respective native language (the majority in Hindko and few in Pushtoon) (Fig 2 and Table 1). Additionally, the free listing technique was employed to record the plant species and their medicinal values. After taking demographic details the ethnomedicinal knowledge of the participants were documented. The reported plants were identified with their vernacular name and collected with the help of local informants in the field. To protect the vouchers from plant pathogens, pests, and fungi the specimens were treated with Mercuric chloride, copper sulphate, and absolute alcohol (2 g mercuric chloride and 10 g copper sulphate dissolved in 1000 ml absolute alcohol) [16, 17]. The plant species were identified using the Flora of Pakistan [18, 19]. The collected plants were identified by Dr. Rizwana Aleem Qureshi, Department of Plant Sciences, Quaid-i-Azam University Islamabad, Pakistan. The botanical names and respective families follow the Angiosperm Phylogeny Group [20]. The Plant List (2010) (http://www.theplantlist.org.), and World flora online (http://www.worldfloraonline.org/). The identified plant specimens were properly labeled, stamped, and given voucher numbers after identification. Finally, they were deposited in the herbarium of Hazara University Mansehra, Pakistan.

**Fig 2:** GIS-based map of the study area depicting targeted localities.

**Table 1:** Description of the visited localities for ethnobotanical data collection.

Community	Latitude (N)	Longitude (E)	Elevation (m)	Population (household)	Ethnicity/Clans
Gandaf	34.1	72.7°	622	2,412	Tanoli, Awan, Syed and Gujjer
Lasan Nawab Sahib	34.37	73.0°	817	2,735	Hindko, Tanoli, Pushtu
Shungli Bandi	34.45	72.96°	1410	1,451	Hindko, Gojri, Tanoli, Pushto
Gali Badral	34.43	73.02°	1502	1,512	Tanoli, Hindko, Pushto, Gojri
Shehargarrh	34.42	73°	1203	2,712	Tanoli, Hindko, Pushto
Beer	34.2	72.9°	839	1,349	
Parrehna	34.3	72.6°	665	3,112	Tanoli, Hindko, Pushto
Chamatti	34.227°	73.034°	849	2025	Tanoli, Awan, Syed and Gujjer
Lasan Thukral	34.2	73°	925	3,678	Hindko, Gojri, Tanoli & Pushto
Pind Kargo khan	34.17°	73.06°	1248	9,375	Tanoli, Awan, Syed and Gujjer
Sherwan	34.19	73.06°	1057	7,815	Tanoli, Hindko, Pushto
Chhar	34.07°	73.09°	1437	69,827	Tanoli, Awan, Syed and Gujjer

### Relative abundance of fodder plants

Kent [21] was followed for the estimation of Relative abundance (RA) (Table 2).

**Table 2:** Abundance categories and scale of reported plants.

Abundance scale	Abundance categories	Coverage of grass species
+	Rare (R)	<5%
1	Occasional (O)	5–20%
2	Frequent (F)	20–50%
3	Common (C)	50–90%
4	Abundant (A)	90–100%


$$\text{Relative}\;\text{abundance}\;\text{of}\;\text{species}=\frac{\text{Total}\;\text{percentage}\;\text{Cover}\;\text{of}\;\text{species}\;\text{in}\;\text{all}\;\text{plots}}{\text{Number}\;\text{of}\;\text{plots}\;\text{estimated}}\times 100$$

### Data analysis

#### Relative frequency of citation (RFCs)

RFC indicates the importance of each species and is calculated based on the frequency of citation ‘FC’ (the number of informants mentioning the use of species. The FC value is divided by the total number of informants participating in the survey (N), without considering the use categories [22]:

RFCs=¼FCs/N

Where FCs is the number of informants who mentioned the use of a plant species and N is the total number of informants.

#### Use Value (UV)

The use-value (UV) is a manifestation of the comparative importance of each plant species employed by the informants in the study range. The value was calculated using the following formula proposed [23]:

UV=ΣU/n

Where, U is the number of use reports quoted by each informant for a given plant species while n refers to the total number of informants interviewed for a given plant [24]. The UV parameter helps to determine which of the plants are most frequently used for a particular purpose. Thus, UV is high when the plant is mentioned by a large number of informants and low when there are few usages cited.

#### Fidelity level (FL)

The fidelity level (FL), is the percentage of informants using a certain plant species for the same purpose, calculated as:

$$\text{FL}\;\left(\%\right)=\left(\text{Np}/\text{N}\right)\;\times 100$$

Where, Np = number of informants that claim use of a plant species to treat a particular illness; N = number of informants that use the plants as a medicine to treat any given disease [25, 26].

### Novelty index (Jaccard index)

Novelty index (Jaccard index (JI)) was calculated by comparing current findings with previously published studies from aligned regions. Following formula was used:

JI=c×100÷a+b−c

where a is the number of species of the area A, b is the number of species of the area B, and c is the number of species common to A and B [27].

### Statistical interference

IBM SPSS 25 version was employed for Descriptive statistical analysis of various qualitative parameters (Frequency and cross tabulation). Furthermore, Pearson Correlation was used to interpret the relationships between quantitative indices i.e. UV and RFC. Hierarchical cluster analysis was also performed for grouping of reported medicinal plants into meaningful groups of high, medium, and low used value plants.

## Result and discussion

### Respondents’ demography and traditional knowledge

A total of 85 participants were interviewed about the ethnomedicinal flora of the Tanawal area in the present work. Most people practice high mountain small level farming and lower hill horticulture, and also rear sheep [28]. Agriculture in most of the area depends on rainfall, and only a small part of the Tanawal is irrigated by diversion of perennial flow water from Siran River and Ichhar Nallah [29]. The major crops grown in the area are maize, rice, tobacco, and wheat. Vegetables and fruits are not common. It is observed that out of all respondents 45.88% came from Mansehra, from Haripur District 21.18%, and District Abbottabad 32.94%. The traditional knowledge regarding medicinal taxa was different based on gender, age, ethnicity, and profession. Interestingly, the female respondents were equally knowledgeable as men in all surveyed areas alike to Voeks [30], who described women, are the reservoirs of traditional knowledge. In the age group between 40–50 years and 60–70 years, female respondents were more knowledgeable than men. In contrast men in the 50–60 year age class were more knowledgeable than women. However, in Mansehra men were more knowledgeable, while women from Abbottabad had higher knowledge. In Haripur showed men held slightly more knowledge were 52% and females were of having 47%. Elderly women (60–70 years) were found equally knowledgeable, but the information provided by them followed a different structure.

This showed that women acquire knowledge later in life. Quick knowledge acquisition and rapid eroding of indigenous knowledge were observed in men with age as compared to women. Reyes-García *et al*. [31] interpreted that elder people retain more knowledge irrespective of gender. But Kainer and Duryea [32] found that women not only demonstrated refined botanical knowledge but were also skilled in plant collection, processing, and management. Our study also showed that women were more proficient in botanical knowledge as compared to men. This may be correlated to women’s engagement with agro-activities, cultural practices, and limited communal life. Men were engaged in outdoor activities and acquired an inclination towards modern medicine, thus losing traditional knowledge.

Similarly, the interviews revealed that the Hindkos (34.12%) and the Tanolis (29.41%) ethnic groups were more knowledgeable ethnobotanically, while Gujjars and Pushtoons had less knowledge (Table 3), although there was no significant difference in medical uses of indigenous plants. This homogenous plant-based knowledge indicates prolong common socio-cultural history. This may also be attributed to similar geophysical localities, settlements, and the local of the Tanawal area. However, some variations in knowledge retention could be perceived in these districts. Mansehra district was first with regard to knowledge, with 91.6% of all plants and uses found there, while Abbottabad and Haripur stood second and third (89.09% and 51.57%.). The retention of indigenous knowledge in Mansehra may be associated with the huge area of mountains, mountain communities, and alpine pastures.

**Table 3:** Respondents’ demography.

**(a) Overview of sampling sites**					
Social variables	Description	Men	Women	No. of people	Percentage
Localities	Haripur District	10	8	18	21.18
	Abbottabad District	13	15	28	32.94
	Mansehra District	21	18	39	45.88
**(b) overall demographic attributes of respondents**					
Sex Ratio	Women	10	9	44	51.76
	Men	11	14	41	48.24
Ethnic groups	Gujjar	17	12	19	22.35
	Tanoli	5	7	25	29.41
	Hindko	15	21	29	34.12
	Pashto	13	12	12	14.12
Age Groups	Between 40–50 years	9	15	36	42.35
	Between 50–60 years	8	12	25	29.41
	Between 60–70	16	13	24	28.24
Education Level	Illiterate	15	7	20	23.53
	Primary	9	5	29	34.12
	Graduate	15	14	22	25.88
	Masters	18	8	14	16.47
Social Livelihoods	Farmers	15	6	29	34.12
	Shepherds	5	4	26	30.59
	Job Holders	10	9	21	24.71
	Wood cutters	11	14	9	10.59

### Taxonomic diversity

We found 66 medicinal plants used by the local inhabitants of the Tanawal area (Table 4). These 66 species belonged to 62 genera and 43 families. Descriptive statistics showed that Fabaceae was the leading family with five species, followed by Euphorbiaceae, Asteraceae, and Solanaceae with four medicinal taxa each. Brassicaceae, Lamiaceae, and Cucurbitaceae presented three species while Berberidaceae, Lythraceae, Malvaceae, and Rosaceae contributed two plant species (Fig 3). The remaining 32 families were monotypic for medicinal taxa of the region. The reported medicinal floral diversity was significant, medical knowledge was widely distributed among the different ethnicities. A taxonomic study might indeed increase details if comprehensive work would be conducted. Due to the rampant urbanization and tourism activities, the infrastructure is rapidly changing and building and highway construction is increasing. Ultimately this causes habitat fragmentation and an increase of plant extraction for sale in the area. It further emphasizes the need for rapid and detailed ethnobotanical surveys to retain ethnoecological knowledge before it is lost forever. The majority of the plants were collected in the wild (80.30%) (Fig 4). The estimation of relative abundance showed some serious concerns about conservation of these indigenous medicinal plants. Results showed only 18% of the species were abundant in study area and that most were occasional (28%) or frequent (24%) (Fig 5). A whole 10% of plants were regarded as rare in the study area (Fig 6). These relative abundance results were alarming and reflected overexploitation of medicinal plants in the study area.

**Fig 3:** The ethnomedicinally dominant families of the study area.

**Fig 4:** Availability status of medicinal plants in the study area.

**Fig 5:** Relative abundance of medicinal plants in the study area.

**Fig 6:** Pictorial view of some valuable medicinal plants of study area (A) *Acacia modesta Wall* (B) *Acacia nilotica* (L.) Delile. (C) *Catharanthus roseus* (Linn.) G. Don (D) *Chenpodium murale* L. (E) *Datura innoxia* Mill (F) *Ricinus communis* L. (G) *Tribulus terrestris* L. (H) *Withania somnifera* L. (I) *Xanthium strumarium* L.

**Table 4:** Documented plants of the Tanawal area Lesser Himalaya, Pakistan.

Family	Botanical name	Local name	Part(s) used	Drug formulation	MA	Ailment(s) cured	S	RA	FC	RFC	UV	FL %	Reporting status with previous studies		
													**NR**	**ARSU**	**ARDU**
Acanthaceae	*Justicia adhatoda* L.	Bhaikarr	Leaves, root, flower,	Decoction & Leaves Smoked	Or	Stimulant, diuretic, tonic, and lice killer	W	O	31	0.365	0.66	36.4	1,2,3,4,5,6,7,8,9,10,11,12,13,14,15,16,17,18,19,20,21	0	0
Acoraceae	*Acorus calamus* L.	Baabchee	Rhizome	Mixture with mustard oil	Or & Top	Children teething, rheumatism	C	R	42	0.494	0.64	49.4	1, 2, 3, 4,5,6,7,8,11,12,13,14,15,16,17,18,19,20,21	0	9, 10
Anacardiaceae	*Schinus molle* L.	kale mirch	Fruit, leaves, bark	Juice, Infusion & Decoction	Or &Top	Used to treat rheumatism; a bark extract infusion is used for diarrhoea, Decoction of ripe fruits are used to treat amenorrhea, bronchitis	C	R	49	0.576	2.3	57.6	1, 2, 3, 4,5,6,7,8,9,10,11,12,13,14,15,16,17,18,19,20, 21	0	0
Apocynaceae	*Catharanthus roseus* (L.) G. Don	Sada bahar	Leaves, flowers	Boiled & Decoction	Or	To control bleeding and to ease sore throats and chest ailments and laryngitis. Also considered for diabetes and as an eyewash for the eyes of infants	C	A	50	0.588	2.4	58.8	1, 2, 3, 4,5,6,7,8,9,10,11,12,13,14,15,16,17,18,19,20,21	0	0
Asteraceae	*Chamaemelum nobile* (L.) All.	Baaobarrang	Leaves	Decoction	Or	Antispasmodic during menstruation, indigestion, and muscle spasms. Also aids with relieving headaches, migraines, and nausea	W	R	42	0.494	0.76	64.4	1, 2, 3, 4,5,6,7,8,9,10,11,12,13,14,15,16,17,18,20,21	0	19
Asteraceae	*Achillea millefolium* L.	Jasifa	Leaves, flower heads	Tea, Crushed dried flowers	Or	Mouth boils, cold and flu and to remove phlegm	W	R	59	0.694	0.58	36.4	1, 2, 3, 4, 5,6,7,9,11,12,13,14,16,17,18,19,20,21	15	8
Asteraceae	*Silybum marianum* (L.) Gaertn.	OOntkattara	Whole plant	Decoction, tea & raw	Or	Used to cure Liver ailments Jaundice	W	F	52	0.612	2.3	61.1	1, 2, 3, 4, 5,9,11,12,13,14,15,17,18,19,20,21	6, 10,16	11
Asteraceae	*Xanthium strumarium* L.	Chottaghokroo	Whole plant	Infusion & Paste	Top	Root is used in earache, fruit used in small-pox.	W	F	48	0.565	2.5	56.6	1, 2, 3, 4, 5,7,8,12,13,14,15,16,17,19,20,21	6	9, 10, 11,18
Berberidaceae	*Berberis lycium* Royle	Sumbal	Leaves, root, bark	Tonic, infusion & tincture	Or & Top	Used in Typhoid, and in C fever. Internal wounds, stomach ache and in diabetes. Externally for wounds, burns & snakebites	W	O	71	0.835	1.26	83.5	1, 2, 3, 4, 5,6.7,8,12,13,14,16,18,20	9,11,15,17,21	10,19
Berberidaceae	*Sinopodophyllum hexandrum* (Royle) T.S. Ying	Bankakri.	Rhizome, Root.	Cooked	Or	Hepatic-stimulant.	W	R	41	0.482	1.1	48.2	1, 2, 4,5,6,7,11,12,13,14,15,16,17,18,20,21	8	3,19
Betulaceae	*Betula utilis* D. Don.	Bhoj pathraa	Leaves, bark	Decoction & Infusion	Or & Top	For treatment of urinary tract infections and in kidney and bladder stones while the bark has been used in the skin infections, the ear, convulsions, wound healing and bronchitis	C	O	37	0.435	2.5	43.5	1, 3, 4, 5,6.7,8,9,11,12,13,14,15,16,17,18,19,21	0	2,20
Brassicaceae	*Brassica campestris* L.	Sarian	Seeds	cooked & raw	Or	Efficient counter-irritant poultice. The oil used as disinfectant and to relieve muscular pains	C	A	80	0.941	1.5	94.1	1, 2, 3, 4, 5,6,7,8,9,10,12,13,14,15,16,17,18,19	11,21	20
Brassicaceae	*Eruca vesicaria* (L.) Cav.	Taramira Jommama	Whole plant	Cooked, Decoction	Or & Top	The oil is used as hair oil to remove dandruff, also used for pain. Cooked plant is considered as Laxative	C	C	78	0.918	1.28	91.7	1, 2, 3, 4,5,6,7,8,9,10,11,12,13,14,15,16,17,18,19,20,21	0	16,20
Brassicaceae	*Sisymbrium irio* L	Khoob-e-kalan	Seeds	Decoction	Or	Seed is used in typhoid, smallpox and cough and in chest debility.	W	A	76	0.894	1.7	91.7	1, 2, 3, 4,5,7,8,12,13,14.15,17,18,19,20,21	6	9, 10, 11,16
Cannabaceae	*Cannabis sativa* L.	Bhang	Leaves, flower heads	Poultice and cooked	Top	The crushed leaves and crushed onions are used for boils in the form of poultice.	W	A	36	0.424	1.5	42.3	1, 2, 3, 4,5,6,7,8,9,10,11,12,13,14,15,16,17,18,19,20,21	0	0
Celastraceae	*Maytenus royleana* (Wall ex MA Lawson) Cufod.	Pataki Kandiari	Seeds and stem	Infusion	Or & Top	Used in digestive problems, The smoke of the seed relieves toothache	C	O	38	0.447	0.7	44.7	1, 2, 3,5,6,7,13,15,17,18,20,21	8,11,12,14	4,9, 10,16,19
Chenopodiaceae	*Chenopodium album* L.	Bathu	Leaves, seeds	Cooked	Or	Useful in peptic ulcers, helminthic and in dyspepsia	W	C	41	0.482	1.76	48.2	1, 2, 3, 4,5,6,7,9,10,11,12,13,15,16,17,18,19,20,21	0	8
Colchicaceae	*Colchicum luteum* Baker.	Qiamat-Gula	Corms	Paste and poultice	Top	Externally applied to relieve neuralgia and itchiness.	W	R	39	0.459	0.6	45.8	1, 2, 3, 4,5,6,7,8,9,10,11,12,13,14,15,16,17,18,19,20,21	0	0
Convallariaceae	*Polygonatum verticillatum* (L.) All.	Noreallam	Leaves, rhizome	Cooked	Or	Rhizome is used in the treatment of pain and considered as diuretic, body tonic and appetizer.	W	R	49	0.576	0.78	57.6	1, 2, 3, 4,5,6,7,8,9,10,11,12,13,14,15,16,17,18,19,20,21	0	0
Cucurbitaceae	*Cucurbita maxima* Duchesne	Kadoo	Fruit	Cooked	Or	Fruits are considered as energetic and have a cooling effect on body	C	C	68	0.8	2.5	80	1, 2, 3, 4,5,6,7,8,9,10,11,12,13,14,15,16,17,18,19,20,21	0	0
Cucurbitaceae	*Citrullus lanatus* (Thunb.) Matsum. & Nakai	Tarbooz	Fruit, seeds	Decoction, powdered & dried seds, Fresh fruits	Or	Increasing urine flow and cleansing the kidneys.	C	A	81	0.953	1.96	95.2	1, 2, 3, 4,5,6,7,8,9,10,12,13,14,15,17,18,19,20,21	11	16
Cucurbitaceae	*Momordica charantia* L.	Karela	Fruit, roots, leaves	Cooked, Poultice, Juice	Or &Top	Purgative, emetic and rubbed in burning sole of feet. The fruit is used in the treatment of diabetes and in hypertension	W	C	81	0.953	3.5	95.2	1, 2, 3, 4,5,6,7,8,9,11,12,13,14,15,16,17,18,19,20,21	0	10
Cupressaceae	*Thuja orientalis* L.	Moor pankh	Leaves, seeds	Boiled & Decoction	Or	Leaves are said as anti-inflammatory and seeds are useful in weakness of body.	C	F	36	0.424	2.5	42.3	1, 2, 3, 4,5,6,9,10,11,12,13,14,15,16,17,18,19,20,21	0	7,8
Dioscoreaceae	*Dioscorea deltoidea* Wall.	Kanees	Rhizome	Cooked	Or	The dried rhizome is fried in desi ghee and used for the treatment of kidney problems.	W	R	33	0.388	3.6	38.8	1, 2, 3, 4, 5,6,7,8,9,11,12,13,14,15,16,18,19,20	17	10,21
Ebenaceae	*Diospyros lotus* L.	Kala Amlok	Fruit, leaves, bark	Infusion	Or	Infusion of the fruit is used as gargle in apathy or stamatitis and sore throat.	W	F	31	0.365	1.12	36.4	1, 2, 3, 4, 5,6,7,8,10,11,12,13,14,15,16,17,18,19,20	9	21
Euphorbiaceae	*Mallotus phillipensis* (Lam.) Müll-Arg.	Kameela	Leaves	Decoction	Or	The plant is considered as anthelmentic and vermifuge.	W	F	37	0.435	2.88	43.5	1, 2, 3, 4,5,6,7,8,9,10,11,12,13,14,15,16,17,18,19,20,21	0	0
Euphorbiaceae	*Phyllanthus emblica* L.	Amla	Fruit, flower, Seeds	Paste, boiled	Or	Exudation from fruit is externally applied on the inflammation of the eye. The fruit is used in pickles and as a jam (fruit preserves) locally termed as Murabba	W	O	67	0.788	1.5	78.8	1, 2, 3, 4,5,6,7,8,10,12,13,14,15,17,18,19,21	16,20	9,11
Euphorbiaceae	*Euphorbia helioscopia* L.	Chatri-dodakDhodal	Roots	Dried powdered form and fresh latex	Top	Milky latex is poisonous, and causes swelling on the skin.	W	A	49	0.576	1.5	57.6	1, 2, 3, 4,5,7,8,9,10,11,12,13,14,15,18,20	6	11,16,17,19,21
Euphorbiaceae	*Ricinus communis* L.	Arund	Leaves, seeds	Poultice and cooked	Or &Top	The bark is used to treat skin inflammations and rashes. A drink of the juice more diluted in water is taken to treat breast tumors and boils	W	A	33	0.388	1.48	38.8	1, 2, 3, 4,5,6,7,8,9,10,11,12,13,14,17,19,21	15,16,18	20
Fabaceae	*Acacia nilotica* (L.) Delile.	Babla, kikar	Bark, Gum	Decoction	Or	Ringworm, urogenital diseases	W	C	37	0.435	1.5	43.5	1, 2, 3, 4,5,6,7,8,11,12,13,14,15,17,18,19	16	9, 10,20,21
Fabaceae	*Acacia modesta* Wall.	Phulai	Bark, Gum	Decoction	Or	Pimples, pneumonia, tonic for woman who gives birth to new baby	W	C	81	0.953	0.78	95.2	1, 2, 3, 4, 5,7,9,10,11,12,13,19,20,21	6,14	8,15,17,18
Fabaceae	*Indigofera heterantha* Brandis	Kainthee	Leaves	Infusion & poultice	Or & Top	Powdered leaves and flowers are used in scabbies and diabetes.	W	F	69	0.812	2.5	81.1	1, 2, 3, 4,5,6,7,8,9,10,11,12,13,14,15,16,17,18,19,20,21	0	0
Fabaceae	*Tamarindus indica* L.	Imlee	Fruit	Infusion, Boiled,	Or	Used in febrile conditions. Fruit is strongly considered as carminative, coolant, antiscorbutic and digestive.	C	F	81	0.953	2.5	95.2	1, 2, 3, 4,5,6,7,8,9,10,11,12,13,14,15,16,17,18,19,20,21	0	0
Fabaceae	*Pongamia pinnata* (L.) Pierre	Sukhchain	Leaves, bark	Decoction	Top	The decoction of leaves and bark is used as bath for fever also used to cure skin ailments and rheumatism.	C	F	74	0.871	2.6	87	1, 2, 3, 4, 5,6.7,8,11,12,13,14,15,19,21	0	9,16,17,18,20
Fumariaceae	*Fumaria indica* (Hausskn.) Pugsley	Pitpaprra	Whole plant	Decoction & tea	Or	Decoction or an infusion of herb is recommended in constipation, leprosy	W	O	35	0.412	1.07	41.1	1, 2, 3, 4,5,6,7,9,10,11,12,13,14,15,16,17,19,20,21	8	18
Hypericaceae	*Hypericum perforatum* L.	balsana	Shoot, flowers	Tea	Or	Green tea is prepared from the leaves, which are considered as stimulant and carminative.	W	R	56	0.659	0.66	65.8	1,4,5,6,7,10,12,13,14,15,16,20	8,2,9,11	3,17,18,19,21,
Juglandaceae	*Juglans regia* L.	Akhroot	Nuts, bark, leaves	Pressed leaves, Dried (bark & fruits), decoction	Or &Top	The leaves are used as lipsticks and for cleaning the teeth. The bark is also useful for the bleeding gums	W	C	67	0.788	1.64	78.2	1, 2, 3, 4, 5,7,8,11,12,13,14,15,16,18,19	6, 10,17	9,20,21
Lamiaceae	*Vitex negundo* L.	Marwaan	Leaves, flowers	Decoction & tincture	Or	Expectorant and are useful in dysentery as a demulcent.	W	F	31	0.365	2.4	49.4	1, 2, 3,6,7,8,10,11,12,13,14,15,16,17,18,19	5,9	4,20,21
Lamiaceae	*Rydingia limbata* (Benth.) Scheen & V. A. Albert	Chitta kanda	Leaves, whole plant	Paste & Poultice	Top	Powder of the plant is mixed with butter and used externally for wounds, also applied on gums to cure tooth ache	W	R	31	0.365	2.1	36.4	5,6,7,8,9,11,12,13,15,16,17,18,19,20,21	3, 4, 10,14,17	1,2
Lamiaceae	*Thymus linearis* Benth.	Ban ajwain	Fruit, whole plant	Infusion, Paste, Tincture	Or & Top	The seeds and flOr shoots are taken internally to cure whooping cough and epilepsy. An Infusion of leaves is used externally for itch and skin eruptions. Seeds are taken as antifebrile and anthelmintic.	W	O	67	0.788	1.8	78.8	1,4,5,7,8,9,12,14	2, 6,10,11,13,15,17,21	3,16,20
Lythraceae	*Punica granatum* L.	Daruna	Fruit, flowers, seeds	Decoction, Paste, Mixture	Or	Used to treat syphilis. Juice used to treat jaundice, diarrhea, nose bleeds and bronchitis.	W	C	74	0.871	1.28	87	1, 2, 3, 4,5,6,7,8,9,10,11,12,13,14,15,16,17,18,19,20	0	21
Lythraceae	*Woodfordia fruticosa* (L.) Kurz	Gul-e- Dhawee	Flowers	Infusion	Or	Dried flowers are astringent, stimulant used to cure stomatitis.	W	R	49	0.576	0.8	57.6	1, 2, 3, 4,5,6,7,8,9,10,11,12,13,14,15,16,17,18,19,20,21	0	0
Malvaceae	*Althaea officinalis* L.	Gul-e-khaira	Roots, leaves, flowers	Decoction & Infusion	Or	Ointment for boils and abscesses, and in a mouthwash for inflammation	C	C	62	0.729	1.3	72.9	1, 2, 3,5,6,7,9,10,11,13,14,15,16,17,18,19,20,21	4,8	12
Malvaceae	*Malva neglecta* Wallr.	Sonchal	Whole plant	Poultice and cooked	Or	A poultice of leaves is useful in relieving sore throats and ophthalmia, and for maturing abscesses.	W	C	64	0.753	1.9	75.2	1, 2, 3, 4, 5,6,7,8,10,11,12,14,15,16,17,18,19,20,21	13	9
Meliaceae	*Azadirachta indica* A. Juss.	Neem	Leaves, flowers	Decoction, infusion & paste	Or &Top	Plant parts are used in dental carries, asthma and in inflammations. Also considered as blood purifier.	W	F	47	0.553	1.4	55.2	1, 2, 3, 4, 5,6,8,10,12,13,14,15,18,19,20,21	7, 11	9,16,17
Moraceae	*Ficus carica* L.	Phagwarr	Fruit, leaves, latex	Paste, Decoction	Or & Top	The fruits emollient pulp helps relieve pain and inflammation, and it has been used to treat tumours, swellings, and gum abscesses.	W	F	37	0.435	1.27	43.5	1, 2, 3, 4,5,6,7,8,9,10,11,12,14,15,16,17,18,19,20,21	0	13
Myrtaceae	*Eucalyptus globulus* Labill.	Gondh	Leaves, shoots	Dried and preessed leaves.	Inhalation	Leaves are used in the form of cigarette for asthma.	W	F	44	0.518	1.3	51.7	1, 2, 3, 4,5,6,7,8,9,10,11,12,13,14,15,16,17,18,19,20,21	0	0
Oleaceae	*Jasminum sambac* (L.) Aiton	Mottia	Root, leaves, flowers	Tea, Paste	Top	Abdominal pains, severe diarrhea	W	F	31	0.365	0.66	36.4	1, 2, 3, 4,5,6,7,8,9,10,11,12,13,14,15,16,17,18,19,20,21	0	0
Orobanchaceae	*Cistanche tubulosa* (Schenk) Wight	Hiran ka khaj	Whole plant	Decoction	Or	Whole plant is used as blood purifier healers, also believe that it is effective in stomach, ache, and diarrhoea and cures sores.	W	R	78	0.918	2	91.7	1, 2, 3, 4,5,6,7,8,10,11,12,13,14,15,16,17,18,19,20,21	0	9
Papaveraceae	*Papaver rhoeas L*.	Laal post	Flowers	Decoction	Or	Effective in cough and in asthma. Also considered it as a pain reliever and in insomnia.	W	C	46	0.541	2.5	54.1	1, 2, 3, 4,5,6,7,10,11,12,13,14,15,16,19,20	8	9,18,17,21
Pinaceae	*Cedrus deodara* (Roxb. ex D. Don) G. Don	Diara	Leaves	Infusion	Or	The leaves are useful in inflammations. The heartwood is emollient, expectorant.	W	O	31	0.365	0.9	36.4	1, 2, 3, 4,5,6,7,8,9,10,11,12,13,14,15,16,17,18,19,20,21	0	0
Platanaceae	*Platanus orientalis* L.	Chanaar	Fruit, leaves, bark	Infusion, Paste, Tincture	Or	The bark boiled in water or in vinegar, and is given for diarrhea and toothache. Bark is very useful in leucoderma and in poisonous biting of stings.	W	C	55	0.647	0.85	64.7	1, 2, 3, 4,5,6,7,8,9,10,11,12,13,14,15,16,17,18,19,20,21	0	0
Poaceae	*Bambusa bambos* (L.) Voss	Bans, babsheer	Leaves, young shoots	Paste, infusion	Or &Top	Young shoot paste is used as antiseptic to treat wounds and is given to treat diabetes. Leaf infusion is given as anthelmintic and febrifuge.	W	F	75	0.882	1.92	88.2	1, 2, 3, 4,5,6,7,8,9,10,11,12,13,14,15,16,17,18,20,21	0	19
Polygonaceae	*Rumex hastatus* D. Don	Khatimbal	Leaves, flowers, shoots	Tonic & paste & tincture	Or & Top	It heals internal tumors, lesions and Ulcers. Also used as digestive aid, and a stomach nerve tonic	W	O	38	0.447	2.1	44.7	1, 3, 4, 5,6,8,11,12,13,14,15,16,19,20	2,9,10	7,18,17,21
Rosaceae	*Pyrus pashia* Buch.-Ham. ex D. Don	Batangi	Fruit	Raw fruits	Or	Taken internally and considered as laxatives and febrifuge.	W	O	42	0.494	3.2	49.4	1, 2, 3, 4,5,6,7,8,11,12,13,14,15,16,17,18,19,20	21	9,10
Rosaceae	*Crataegus songarica* K. Koch	Batsanglee	Berries	Extract, Decoction	Or	Cardiac tonic. Also having cholesterol level lowering activities	W	O	31	0.365	2.1	36.4	1, 2, 3, 4	0	0
Rutaceae	*Citrus limon (L*.*) Osbeck*	Nimbu	Fruit, leaves	Juice, Decoction, Infusion, Paste	Or &Top	Helps in reduction of fats. Rind of ripe fruit is stomachic and carminative. Juice of ripe fruit is refrigerant.	W	F	80	0.941	2.6	94.1	1, 2, 3, 4,5,6,7,8,9,10,11,12,13,14,15,16,17,18,19,20,21	0	0
Salicaceae	*Casearia tomentosa* Roxb.	Chilla,	Fruit, bark	dried fruits	Or	fruit is a fish poison which can affect human health when intake that poisoned fish	W	O	47	0.553	0.6	55.2	1, 2, 3, 4,5,6,7,8,9,10,11,12,13,14,15,16,17,18,19,20,21	0	0
Solanaceae	*Datura innoxia* Mill.	Tatulaa	Seeds, leaves, flowers	Paste, tea, Smoked	Inhalation	Datura is often mixed with cannabis and this mixture is smoked to relieve asthma and rheumatism. Usd as Antilice	W	O	41	0.482	2.4	48.2	1, 2, 3, 4,5,6,7,8,9,10,11,12,13,14,15,16,17,18,19,21	0	20
Solanaceae	*Hyoscyamus niger* L.	Dewanaphang	Leaves and seeds	Dried seeds	Or	The seeds are chewed for relieving toothache.	W	O	50	0.588	1.4	58.8	2, 3, 4,5,6,7,9,10,11,13,15,16,17,18,19,20,21	1	12,14
Solanaceae	*Withania coagulans* (Stocks) Dunal	Asganth Paneer band	Fruit, twigs	Infusion, Cooked,	Or &Top	The fruits are reported to be sedative, emetic and diuretic. They are useful in chronic disorders of liver. The twigs are chewed for cleaning teeth and toothache	W	O	55	0.647	3.3	64.7	1, 2, 3, 4,5,6,7,8,9,10,11,12,13,14,15,16,17,18,19,21	0	20
Solanaceae	*Withania somnifera* (L.) Dunal.	Asganth	Roots	Decoction, Paste	Top	A paste of the roots and bruised leaves applied to carbuncles, ulcers and painful swelling	W	O	37	0.435	2.4	43.5	1, 2, 3, 4,5,6,7,8,11,12,13,14,15,18,19,21	16,17	9,10,20
Thymeleaceae	*Daphne mucronata* Royle	Kutilaal	Whole plant	Decoction	Or	The plant is cooling, alterative and anthelmintic	W	O	72	0.847	1.13	84.7	1, 3,4, 5,6,7,8,11,12,13,14,15,16,17,18,19,20,21	10	2
Violaceae	*Viola canescens* Wall.	Banafsha	Flowers, roots	Infusion	Or	An infusion of flowers with almond oil is a gentle laxative for children and helps to soothes irrigative cough	W	O	71	0.835	2.6	83.5	1, 2, 3, 4,5,6,7,11,12,13,14,15,16,17,19,20	8,18,21	9
Vitaceae	*Vitis vinifera* L.	Angoor	Fruit, leaves	Decoction, Paste	Or &Top	To relieve the discomfort of varicose veins. Infusion of leaves applied as a wash, eye drops or eye washes, very useful in rheumatism	W	F	78	0.918	2.2	91.7	1, 2, 3, 4,5,6,7,8,9,10,11,12,13,14,15,17,18,19,20,21	0	16
Zygophyllaceae	*Tribulus terrestris* L.	Bhakraa, Ghokru	Fruit, leaves	Cooked	Or & Top	For spermatorrhoea and general debility	W	O	35	0.412	2.7	41	2,4,5,6,7,12,13,14,15,16,17,18,19,20	10	1,3,9, 11,21

1. [34]; 2. [50]; 3. [1]; 4. [51]; 5. [52]; 6. [45]; 7. [60]; 8. [53]; 9. [38]; 10. [54]; 11. [40]; 12. [55]; 13. [56]; 14. [44]: 15. [43]; 16. [57]; 17. [42]; 18. [58]; 19. [59]; 20. [39]; 21. [41].

### Part(s) used, drug formulation and administration mode

Based on descriptive statistics leaves (43.28%) were the predominantly used medicinal plant part, followed by whole plant and fruits (both 14.92%). Flowers (13.67%, seeds, roots, bark (10.44%) and gum (2.67%) were less commonly used (Fig 7). The most common recipe of drug preparation was decoction i.e. 21 species (31.15%). However, infusion and paste formulations were also commonly used (paste 12 species, 17.21%; and infusion 11 species, 18.83%). The remaining plants were used cooked form (9 species 13.34%), as a poultice (5 species, 7.46%), tea (5 species, 7.46%), and raw (4 species, 5.97%). Local people of the Tanawal area preferred oral administration (56.1%). However, 28% of medicinal plants accounted for both oral and topical applications (Figs 8 and 9).

**Fig 7:** Depiction of parts used of medicinal plants.

**Fig 8:** Percentage of the mode of drug administration.

**Fig 9:** Percentage of the mode of drug administration.

### Medicinal plants versus disease(s) cured

A total of 50 health disorders recorded in the study area were grouped in 15 categories. These categories were evaluated for the total number of taxa used. It was revealed that maximum species were used to treat gastrointestinal disorders (13 species), dermal problems (12 species), respiratory tract ailments (9), and hepatic disorders (8). Seven species were used for musculoskeletal problems and general body debility, while six species were used for dental disorders, as a laxative, as a diuretic, and for urinary tract infection. Similarly, for the treatment of diabetic ailments and anti-inflammatory five species were used while for renal problems, ophthalmic disorders, and sore throat four species were used. Gastrointestinal (GIT) disorders (i.e. constipation, indigestion, gastric trouble, dysentery, acidity, and stomach ulcer), skin diseases (pimples, pustules, and ringworm), respiratory tract infections (bronchitis, asthma, pneumonia), and musculoskeletal ailments were the common health problems. The prevalence of gastrointestinal (GI) disorders may be attributed to poor available hygiene. The harsh and hostile weather might contribute to getting respiratory infections, and the limited sanitary facilities might contribute to intestinal problems. The painstaking activities for survival in this difficult topography might lead to cramps and orthopedic disorders. Intestinal ailments, skin-related diseases, and problems concerning the digestive system were among the highest medical problems reported categories in the Tanawal community. These recurrent health issues may be attributed to harsh weather, lack of hygiene, and poor food selection [33, 34]. Other common medicinal uses categories mentioned by respondents included the muscular-skeletal system, urinary system, and general body tonic (Fig 10).

**Fig 10:** Categories of diseases of the study area and number of plants used.

### Statistical data analysis

Homogeneity in the traditional knowledge was evaluated using quantitative indices i.e. Relative Frequency of Citation (RFC). RFC indicates the significance and status of a particular medicinal plant in the targeted human community [35]. Higher RFC values indicate the retention and smooth transmission of traditional knowledge among local people [36]. In our study the highest RFCs were calculated for *Acacia modesta*, *Citrullus vulgaris*, *Tamarindus indica* and *Momordica charantia* with 81 each. Some other species had high values, e.g., *Brassica campestris* (80), *Citrus limon* (80), and *Eruca sativa* (78). This indicates the stability of traditional therapeutic information regarding highly cited species. *Jastacia adhatoda*, *Vitex negundo*, *Jasminum sombac*, *Diospyrus lotus*, *Cedrus deodara* and *Otostegia limbata* scored low RFC values indicating their least medicinal importance.

To assess the relative importance on the uses of reported plants Use Value was used. Use value (UV) is an index widely used to quantify the relative importance of useful plants [37]. The Use Value (UV) ranged from 0.66 (Colchicum luteum) to 3.6 (*Dioscorea deltoidea*. *Withania coagulans* (3.3), *Momordica charantia (3*.*5)*, *Silybum marianum*, *and Pyrus pashia* also reported with high UV values. The Pearson correlation between UV and RFC reflected a positive correlation. However, the coefficient value was quite low (0.0316) which showed that these two indices are nearly independent to each other in concern to the ethnobotanical knowledge of the Tanawal community. This might be interpreted by the fact that RFC is only the indicator of the familiarity or popularity of a particular plant in the study area. Abundance and availability in the wild could be possible reasons for their popularity in the study area. RFC does not indicate the diversity in plant utilization from the medicinal perspective and it can only be predicted by UV application.

The Pearson correlation between UV and RFC reflected a positive correlation. However, the coefficient value was quite low (0.0316) which showed that these two indices are nearly independent to each other in concern to the ethnobotanical knowledge of the Tanawal community. This might be interpreted by the fact that RFC is only the indicator of the familiarity or popularity of a particular plant in the study area. Abundance and availability in the wild could be possible reasons for their popularity in the study area. RFC does not indicate the diversity in plant utilization from the medicinal perspective and it can only be predicted by UV application (Fig 11).

**Fig 11:** Pearson correlation between RFC and UV.

The Fidelity Level (FL) is the percentage of informants claiming the use of a particular plant species for the same major purposes or requirements, was also determined for the most frequently reported diseases or ailments. The calculation revealed that 28 (41.79%) species had FL values below 50, while 39 (58.20%) had higher FL values. The FL values ranged from 36.4 to 95.2. The taxa securing highest values were *Momordica charantia*, *Tamarindus indica*, *Acacia modesta* and *Citrullus lanatus* with 95.2. *Rydingia limbata*, *Crataegus songarica*, *Jastacia adhatoda* and *Diospyrus lotus* were the taxa securing lowest Fl values. FL% basically reflects the significance of plant for particular use. Multiple ethnomedicinal studies suggested that plants with highest FL% can be considered as the most useful.

#### Cluster analysis

Based on UVs, the total 66 reported medicinal plants were clustered into 3 groups. Cluster 1 comprised of those plants that had lower UVs (0.66–1.13), plants of cluster 2 possessed comparatively higher UVs (2.3–2.7), whereas, plants of cluster 3 (*Momordica charantia*, *Dioscorea deltoidea*, *Pyrus pashia*, *Withania coagulans* had the highest reported UVs (3.2–3.6) (Fig 12).

**Fig 12:** Showing the clusters based on UVs.

#### Cross tabulation between three clusters and relative abundance (RA)

Cross tabulation between three clusters and relative abundance (RA) reported that the relative abundance of plants declines by the increase of their UVs. It can be said that the higher the utilization aspect, the lower the relative abundance in a particular study area. It can be observed that among the 4 plants of cluster 3 (with uppermost UVs), none of the plants was reported as abundant in the study area. However, in cluster 2, only 2, and in cluster 1 (lowermost UVs), 5 were reported as abundant in the study area. As the utilization of plants lowered the probability of their abundance increases simultaneously (Table 5).

**Table 5:** Relative abundance * cluster no. cross tabulation.

Count					
		Cluster no.			Total
		1	2	3	
**Relative Abundance**	Abundant	5	2	0	7
	Common	9	2	1	12
	Frequent	5	11	0	16
	Occasional	10	7	2	19
	Rare	8	3	1	12
Total		37	25	4	66

### Novelty index

The current study results were compared with ethnobotanical literature to draw novel aspects of the study. The similarity index was calculated using the Jaccard Index (JI) (. Documented 66 ethnomedicinal plants of this study had been cross verified in the 21 published articles that had similar geographic or climatic conditions (Table 4). In the current study, the JI values ranged from16.77 to 0.98 (Table 6). The highest values have been reported by the Gokand Valley of District Buner [38] followed by the Banda Daud Shah in Karak [39], Karamar Valley [40], Patriata, and New Murree [41] and Charmang village in Bajur [42] i.e. ≥ 11. A higher JI value reflects the similarity in vegetation types of two areas due to similar geographic or climatic conditions [43]. The lowest JI (2.15) was calculated in comparison to study of Kayani *et al*. [44] (Alpine and sub-Alpine regions). The current study showed a greater resemblance with data of Manoor valley [45] (25.92%). This indicates that although Gokand Valley and Tanawal share a similar flora, however, their usage patterns are more analogous to Manoor Valley. These resemblances and variations arise due to the ecological [46] historical [47], organoleptic [48], and phytochemical differences [49] across the regions. The current study also reported 16 medicinal plants which have been rarely documented for their medicinal use in the studied ethnomedicinal literature i.e. *Althea officinalis*, *Plantanus orientalis*, *Jasminum sombac*, *Maytenus royleana*, *Cucurbita maxima*, *Phyllanthus emblica*, *Citrullus vulgaris*. *Polygonatum verticilliatum*, *Caseria tomentosa*, *Cistanche tubulosa*, *Bambusa arundinacea*, *Schinus molle*, *Tamarindus indica*, *Pongamia pinnata*, *Citrus limon* and *Catharanthus roseus*.

**Table 6:** Jaccard index of the medicinal flora.

Citation	Study area	Province	Np	NPSU	NPDU	TPCBA	PRAA	PRSA	PPSU	PPDU	JI
Abbas et al. (2016)	Tormik Valley	GB	63	1	2	3	60	62	1.59	3.17	2.40
Shoaib et al. (2017)	Lowe kaghan Valley	KPK	46	3	3	6	40	59	6.52	6.52	5.71
Abbas et al. (2017)	Shigar Valley	GB	84	1	4	5	79	60	1.19	4.76	3.47
Bano et al. (2014)	Skardu valley	GB	50	1	2	3	47	62	2.00	4.00	2.68
Majid et al. (2019)	Lesser himalayan	KPK	38	1	0	1	37	64	2.63	0.00	0.98
Rahman et al. (2019	Manoor Valley	KPK	27	7	0	7	20	58	25.93	0.00	8.24
Abbasi et al. (2013b)	Lesser Himalayan	KPK	45	2	2	4	41	61	4.44	4.44	3.77
Khan et al. (2013)	Naran valley	KPK	101	7	4	11	90	54	6.93	3.96	7.10
Sulaiman et al. (2020)	Gokand Valley	KPK	109	9	16	25	84	40	8.26	14.68	16.78
Ahmad et al. (2011)	Tehsil Kabal	KPK	140	7	10	17	123	48	5.00	7.14	9.04
Khalid et al. (2017)	Karamar Valley	KPK	63	7	6	13	50	52	11.11	9.52	11.30
Tariq et al. (2019)	Ione valley	KPK	35	1	2	3	32	62	2.86	5.71	3.09
Khan et al. (2014)	Haripur	KPK	10	2	1	3	7	62	20.00	10.00	4.17
Kayani et al. (2015)	Alpine and sub alpine region	KPK	125	3	1	4	121	61	2.40	0.80	2.15
Farooq et al. (2019)	Dhirkot	AJK	140	4	1	5	135	60	2.86	0.71	2.50
Adnan et al. (2014)	northwest Pakistan		107	5	9	14	93	51	4.67	8.41	8.861
Abidullah et al. (2019)	Charmang village, Bajur	KPK	64	6	7	13	51	52	9.38	10.94	11.207
Ullah et al. (2020)	Sheen Ghar Valley, Dir	KPK	51	2	7	9	42	56	3.92	13.73	8.411
Ahmad et al. (2017)	Neelum valley	AJK	50	0	7	7	43	58	0.00	14.00	6.481
Murad et al. (2013)	Banda Daud Shah, Karak	KPK	58	1	12	13	45	52	1.72	20.69	11.818
Ahmed et al. (2013)	Patriata and New Murree	KPK	93	5	11	16	77	49	5.38	11.83	11.268

**Key:** GB-Gilgit Baltistan; KPK-Khuber Pakhtoon kha; AJK-Azad Jamu Kashmir; Np number of participants, NRPs number of reported plant species, NPSU number of planst with similar uses, NPDU number of plants with different uses, TPCBA total plants common in both area, PRAA Plants reported in aligned areas, PRSA Plants reported only in study area, PPSU percentage of plant with similar uses, PPDU percentage of plant with different uses, JI Jaccard index.

## Conclusion

Current ethnobotanical investigation showed that the people of the Tanawal area retain substantial indigenous knowledge. The people of all ethnic groups keep and transmit their information related to plants irrespective of gender, locality, and ethnicity. But the old people seem to be the real caretaker of this knowledge. They use a considerable number of medicinal taxa to treat their ailments as a basic remedial source. However, a rapid trend in tourism and infrastructural development causes direct habitat destruction in the area. Moreover, broad-scale medicinal plant extraction, deforestation, and grazing are also potential human-made threats to medicinal species. These factors could be detrimental for both phyto-medicinal taxa and associated knowledge. The establishment of medicinal plant nurseries and their cultivation will be an effective measure for their conservation. On the other hand, the species which were identified as of great importance and constancy in the focused communities could be investigated against their reported therapeutic potentials. The study is a preliminary survey and maybe a potential literary contribution for local researchers, conservationists, and policymakers.

## Supporting information

S1 File Questionnaire employed in study. (PDF)

S1 Table Main table showing all collected ethnobotanical data. (XLSX)

S2 Table RFC calculations. (XLSX)

S3 Table UV calculations. (XLSX)

S4 Table FL calculations. (XLSX)

S5 Table SPSS data set. (SAV)
